The article "Quantifying Significance of Topographical Similarities of Disease-Related Brain Metabolic Patterns" was published in 2014. Journal: PLoS One.

# Quantifying Significance of Topographical Similarities of Disease-Related Brain Metabolic Patterns

**DOI:** 10.1371/journal.pone.0088119

**Published:** 2014-01-31

**Authors:** Ji Hyun Ko, Phoebe Spetsieris, Yilong Ma, Vijay Dhawan, David Eidelberg

**Affiliations:** Center for Neurosciences, The Feinstein Institute for Medical Research, North Shore-Long Island Jewish Health System, Manhasset, New York, United States of America; University of Toronto, Canada

## Abstract

Multivariate analytical routines have become increasingly popular in the study of cerebral function in health and in disease states. Spatial covariance analysis of functional neuroimaging data has been used to identify and validate characteristic topographies associated with specific brain disorders. Voxel-wise correlations can be used to assess similarities and differences that exist between covariance topographies. While the magnitude of the resulting topographical correlations is critical, statistical significance can be difficult to determine in the setting of large data vectors (comprised of over 100,000 voxel weights) and substantial autocorrelation effects. Here, we propose a novel method to determine the p-value of such correlations using pseudo-random network simulations.

## Introduction

Spatial covariance analysis of scans of resting cerebral function provides a useful way to characterize specific network abnormalities in a variety of neurodegenerative disorders [1]–[5]. This approach has been particularly valuable in elucidating the systems-level changes in cerebral function that underlie hypokinetic movement disorders such as Parkinson’s disease (PD) [1], [5], as well as atypical variant conditions such as progressive supranuclear palsy (PSP) and multiple system atrophy (MSA) [6], [7]. Moreover, spatial covariance patterns can be used in combination to differentiate these clinically similar conditions based upon their characteristic metabolic topographies [8], [9]. Despite consistent evidence that the expression of these disease-related covariance patterns is independent in individual subjects, scant information exists concerning the actual relationship of the topographies between any two topographies.

To assess similarities and differences between relevant functional networks, we developed a computational algorithm in which voxel weights (i.e., the regional loadings on principal component (PC) patterns) on two spatial covariance topographies are cross-correlated by computing the Pearson product-moment correlation coefficient [10]–[12]. For example, in a recent study we analyzed topographical relationships between the abnormal PD-related metabolic covariance pattern (PDRP) [4], [13] and the normal movement-related activation pattern (NMRP) [12], [14] that is deployed by both PD and healthy subjects during motor performance [15]. Intuitively, the correlation between the voxel weights on the two topographies is at best modest (r^2^ = 0.074). Nonetheless, the p-value associated with the computed correlation coefficient exceeded the threshold for rejecting the null hypothesis that the two topographies were not different (p<0.001). In all likelihood, the statistical significance of the correlation between the voxel loadings on the two covariance patterns was exaggerated by spatial autocorrelation. The source of the autocorrelation comes from regional intrinsic connectivity and remote functional connectivity, which may be also elevated in the preprocessing procedures such as spatial normalization and smoothing. To adjust for such effects in the assessment of correlations between very large data vectors (>100,000 voxel pairs), we simulated 1,000 pseudo-random volume pairs containing a degree of autocorrelation (measured by Moran’s I [16]) that was similar to those measured for each of the actual pattern topographies [cf. 17]. This method allowed for the non-parametric computation of an adjusted p-value with which to assess the significance of the observed topographic correlations. To demonstrate this approach, we used it to evaluate topographic inter-relationships between the PDRP and previously characterized metabolic patterns associated with MSA and PSP, the two most common parkinsonian “look-alike” conditions. In addition, we also compared PDRPs derived from five different PET centers from USA, Netherlands, China, India and South Korea.

## Methods

Imaging protocols and pattern characterization procedures are described elsewhere [1], [4], [6], [7], [13]. A tutorial on the use of this covariance approach has appeared recently [18].

### Topographical Correlation

Similarities/differences between the PDRP [13], MSA-related pattern (MSARP) [6], [7] and PSP-related pattern (PSPRP) [6], and PDRPs from four different countries (i.e., USA, Netherlands, China and India) [5] were evaluated by computing the percent of the overall variance shared (r2) between the non-zero voxel weights on each pair of topographies [10], [11], [15]. Voxels from each pattern image were formatted into a single vector by appending successive rows in each plane of the image. The two vectors were then entered into the MATLAB statistical routine “corr” to calculate the correlation coefficient (r).

### Determining the Window Size of Local Moran’s I for Estimating Autocorrelation

To estimate the spatial autocorrelation within each of the disease-related metabolic patterns, we computed a global Moran’s I for the whole brain [16], [19]. First, local Moran’s I is computed at each voxel within a moving window thereby representing spatial autocorrelation within the pre-defined area centering at each voxel, then it was averaged across the whole brain (i.e., global Moran’s I) [19]. No consensus exists regarding the optimal window size for local Moran’s I in neuroimaging studies. We, therefore, empirically determined the window size on this parameter that best predicted the observed topographical correlation in spatially autocorrelated volume-pairs. This was accomplished in a separate simulation study in which 300 pseudo-random volume pairs were selected. Each volume was comprised of 116 regions defined by the automated anatomical labeling (AAL) algorithm [20]. Within a given volume, each region was assigned pseudo-random numbers (Gaussian distribution with mean of zero and standard deviation of one). Gaussian noise (mean of zero and standard deviation of 0.05) was added to each volume and smoothed with a box filter of increasing kernel size (3×3×3 to 23×23×23 voxels). The local Moran’s I was estimated for each voxel within each 2D slice then averaged over the brain mask identified with AAL. The global Moran’s I for 3,600 volumes ( = 600 pseudorandom volumes × 6 different box filters) was estimated with different window sizes (W) [of local Moran’s I] (3×3, 9×9, 15×15, 21×21, 27×27, 33×33, 45×45, 51×51, 57×57 voxels) (Figure 1). The 1,800 volume-pairs were then vector-transformed and tested for topographical correlation described above. Multiple regression analysis was employed to determine the W for which the average local Moran’s I of the simulated pairs was most closely related to the increase in topographic correlation induced by the box filter. The Akaike Information Criteria (AIC) was utilized to identify the best model fit. The selected W-value was used to compute local Moran’s I in the subsequent simulation studies (Table 1).

**Figure 1:** Schematic diagram of the simulation study. The stimulation was conducted to determine the Window size of Moran’s I that best reflected the inflated topological correlation of the two simulated networks. (**A**) 300 pseudo-random volume-pairs were generated, then box filters were applied to each volume with six different kernel sizes (3×3×3, 7×7×7, 11×11×11, 15×15×15, 19×19×19, 23×23×23). Then, the global Moran’s I of 1800 volume-pairs (300 original volume-pairs×6 different box filters) was estimated with varying window (W) size (3×3, 9×9, 15×15, 21×21, 27×27, 33×33, 45×45, 51×51, 57×57). The volume-pairs were then vector-transformed and tested for voxel-by-voxel Pearson’s correlation (topographical correlation). Multiple regression was utilized to test if the global Moran’s I significantly predicted the box-filtering-induced elevation of topographical correlation. The window size of the Moran’s I (W) that gave the best prediction of the topographical correlation from the global Moran’s I was identified using AIC. (**B–D**) The inflated topographical correlation was observed regardless of the W of Moran’s I while the best prediction resulted when the W of Moran’s I was 51 (lowest AIC).

**Table 1:** The result of multiple regression: |r| = MI*b1+Z*B.

	Window size of local Moran’s I (W)									
	3×3	9×9	15×15	21×21	27×27	33×33	39×39	45×45	51×51	57×57
**b1**	0.764	0.125	0.245	0.318	0.395	0.474	0.543	0.608	0.679	0.757
**se**	1.421	0.342	0.205	0.158	0.136	0.125	0.122	0.125	0.135	0.151
**t**	0.538	0.365	1.199	2.014	2.907	3.778	4.443	4.851	5.044	5.028
**p**	0.591	0.716	0.231	0.044	0.004	1.64E-04	9.54E-06	1.36E-06	5.13E-07	5.55E-07
**AIC**	−5661.9	−5661.4	−5659.8	−5659.7	−5662.2	−5666.2	−5670.2	−5672.9	−5673.8*	−5673.1

* The lowest AIC value.

r: topographical correlation (Pearson’s correlation of the voxel weights of the two simulated patterns; MI: global Moran’s I; b1: coefficient of multiple regression of avgMI; Z: random effects dummy variables for 300 volume-pairs; B: coefficient for random effects; se: standard error of b1; AIC: Akaike Information Criteria for the whole model fit.

### Estimating p-value for Topographical Correlation of the Known Spatial Covariance Patterns

For each comparison between two patterns (e.g., PDRP vs. MSARP; PDRP vs. PSPRP; PDRP (USA) vs PDRP (China)), 1,000 pseudo-random volume-pairs were simulated in the same manner with AAL-based phantom brain described above. The pseudo-random volumes were smoothed with a box filter. The kernel size of the box filter was increased from 3×3×3 to 23×23×23 until the spatial autocorrelation for each volume achieved a value for average local Moran’s I that was similar to that determined for the given spatial covariance pattern. In each iteration, the correlation of the generated volume pairs were evaluated; this simulation procedure was repeated 1,000 times. We then calculated the rank of the r^2^ value that corresponded to the magnitude of the correlation (r^2^) that was directly observed between the two voxel weight vectors. For example, in the correlation between the PDRP and PSPRP voxel weights, 459 volume-pairs exhibited correlations of magnitude greater than the observed r^2^ value of 0.011 (i.e., topographical correlation r^2^ between PDRP and PSPRP), which corresponded to p = 0.459, which was not statistically significant. Because of the multiple pairwise comparisons that were performed across topographies (i.e., PDRP, PSPRP and MSARP, and four different PDRPs), we applied the Bonferroni correction to the resulting p-values.

### Post-hoc Analysis for Evaluating Regional Differences

After quantifying overall topographical similarity between two patterns, one can directly examine the regional differences between the two patterns by simple arithmetic subtraction. The statistical significance of the regional difference is evaluated by permutation test, if 1) source images are available and 2) the patterns are derived in the same manner. Subjects were swapped randomly between two data samples, and the covariance patterns were re-derived in each swapped data set. Difference maps between the swapped pattern-estimates can generate voxel-wise null distributions on which the difference in the point estimates can be judged for statistical significance. In other words, the real difference of region weights can be ranked in permuted differences, then the non-parametric p-value may be estimated, e.g., if the region weight difference is ranked at top 20^th^ out of 1,000 permutation, the p-value is estimated as p = 0.04 (two-tailed). Here, we compared the historical PDRP from USA [13] and the PDRP derived from a new cohort of 18 PD patients and 16 controls from South Korea. The patients in the USA were off anti-parkinsonian medication for >12 hours when they were scanned with FDG-PET while Korean patients were on their regular medication. In order to test if the topographical difference between the two PDRPs stemmed from medication status, the resulting difference-map was again tested for topographical correlation with T-map estimated by comparing 15 independent PD patients who were investigated during levodopa infusion compared to off-state (paired t-contrast) [21].

We used SPM5 software (http://www.fil.ion.ucl.ac.uk/spm/software/spm5/) for preprocessing and the statistical tool box in Matlab 7.7.0 for the simulations and statistical tests.

## Results

### Autocorrelation Inflates Topographic Inter-relationships between Covariance Patterns

As predicted, voxel-level correlations between the two simulated volumes varied with global Moran’s I (Table 1; Figure 1). Thus, the presence of autocorrelation within each network volume artificially increased the degree of correlation that was observed across the two network volumes. Increases in the absolute topographical correlation (|r|) were most closely related to average local Moran’s I for W = 51×51 (Table 1). This window was therefore selected for use in the simulation studies.

### Topographical Correlation between Known Disease-related Networks

The voxel-level topographical correlation between PDRP and either parkinsonian syndrome-related patterns were not significant (p>0.05) (Table 2). Although it did not survive the correction for multiple comparisons, a moderate-level of topographical similarity was observed between PSPRP and MSARP. On the contrary, PDRPs from the four different countries were significantly correlated with each other (p<0.001) (Table 3).

**Table 2:** Voxel-wise topographical correlation (r) of the PD, MSA and PSP-related brain networks.

	PDRP	PSPRP	MSARP
PDRP	.	0.1031 (p = 0.459)	−0.2806 (p = 0.075)
PSPRP	0.1031 (p = 0.459)	.	0.3549 (p = 0.021)
MSARP	−0.2806 (p = 0.075)	0.3549 (p = 0.021)	.

* p<0.05 after Bonferroni correction for multiple comparisons (3 comparisons: p<0.0167).

The p-value is empirically calculated based on the rank of r^2^-value in 1,000 simulations.

**Table 3:** Voxel-wise topographical correlation (r) of the PDRPs from 4 different countries.

	PDRP (USA)	PDRP (Netherlands)	PDRP (China)	PDRP (India)
PDRP (USA)	.	0.7299* (p<0.001)	0.8529* (p<0.001)	0.8558* (p<0.001)
PDRP (Netherlands)	0.7299* (p<0.001)	.	0.7307 (p<0.001)	0.7482* (p<0.001)
PDRP (China)	0.8529* (p<0.001)	0.7307* (p<0.001)	.	0.8265* (p<0.001)
PDRP (India)	0.8558* (p<0.001)	0.7482* (p<0.001)	0.8265* (p<0.001)	.

* p<0.05 after Bonferroni correction for multiple comparisons (6 comparisons: p<0.00833).

The p-value is empirically calculated based on the rank of r^2^-value in 1,000 simulations.

### Regional Differences between PDRPs with Different Medication Status

The topographical correlation between PDRPs derived from USA and South Korea was significant (r = 0.6999, p<0.001) but it was slightly lower than other between-PDRP correlations (r>0.7299; Table 3). The variances-not-accounted-for (i.e., 51%) may be explained by different scanner type, ethnicity, inter-individual differences and medication status. Here, we had an independent set of 15 PD patients who underwent FDG scans on and off levodopa [6]. Standard SPM analysis with paired-design [22] produced a t-map (Figure 2A) which then again compared for topographical similarity with the independently generated difference map (i.e., regional difference between PDRPs from USA vs. South Korea, Figure 2B). The result was significant according to the proposed p-value adjustment (r = 0.4228, p<0.001). This result proposes that the regional difference-map (Figure 2B) reflected in part the differences in medication status between the two PDRPs.

**Figure 2:** Regional differences of two covariance patterns. (**A**) Standard SPM analysis with paired t-test design for ON vs. OFF medication with 15 PD patients. (**B**) The PDRP derived from USA (off-medication) was subtracted from the PDRP derived from South Korea (on-medication). The resulting difference map is z-scored. Only the voxels that were reliable in permutation test were shown (p<0.05, 1,000 permutation). The topography of within-subject differences in medication status (A) was significantly correlated with between-group network differences (B) (r = 0.4228, p<0.001). Likewise, key regions of hypometabolism (e.g., M1, cingulate, cerebellum, putamen) and hypermetabolism (e.g., precuneus) were similarly shown.

## Discussion

As predicted, increasing the autocorrelation within each simulated brain network inflated the voxel-wise topographical correlation between the two independently generated brain networks (Figure 1, Table 2). Thus, p-values computed for each topographical correlation need to account for such potential false positive correlations. Indeed, significant correlations were not evident between PDRP and either of the two atypical topographies. This underscores the substantial pathological differences that exist between idiopathic PD and both MSA and PSP [6], [7], [9]. Interestingly, a marginal similarity was seen for the PSPRP and MSARP topographies (r = 0.35, p = 0.02), perhaps reflecting an overlap in frontal lobe volume loss in the two syndromes [6], [7], [9]. As predicted, the topographical correlation among the four PDRPs from different countries remained to be significant (p<0.001; Table 3).

The proposed methodology may be applicable to a wide range of network analyses. For example, in the exploding literatures on rest-state default mode networks (DMN), researchers have been naming their brain networks as DMN based on their subjective visual inspection [cf. 23]. The proposed method supplies researchers ability to employ null hypothesis testing in determining the similarities of given network patterns compared to the baseline patterns previously described elsewhere [e.g., 24].

In addition, we also examined a method that directly comparing the regional differences between the two patterns. We showed that the simple subtraction of PDRPs derived in different medication status (Figure 2B) was significantly correlated with within-subject differences in medication status (Figure 2A). However, the regional differences between two patterns can only be evaluated if source images are available and if the two patterns are derived in the same manner. This post-hoc analysis is not suitable for locating the regions that are similar between the two patterns, e.g., negative findings may stem from either the similarity of the two patterns or instability of the region estimates.

### Limitation

The autocorrelation (i.e., Moran’s I) was estimated within each slice of volumes, then averaged across the whole brain for computational simplicity and efficiency. This procedure may, however, neglect autocorrelation effects in the dorsal-ventral axis. Thus, some false positive correlations remain possible, even with this method. That is, using the current approach, simulated pseudo-random brain networks may exhibit less autocorrelation than actual covariance topographies, resulting in greater “significance” (i.e., lower p-values) for correlations of specific volume-pairs. This inflation of correlational significance may be offset to some degree by implementing a multiple comparisons correction for the different volume pairs analyzed (see Table 2).

For computational speed we chose to simulate only 1,000 volume-pairs for each topographical correlation study. Even so, the calculations took 1–4 weeks to perform, depending on the degree of autocorrelation estimated for the various patterns (Intel(R) Core(TM) i7-2600 CPU 3.40 GHz, 8.00 GB RAM, 64-bit Windows 7 Professional). Clearly, further research to optimize the computational process is warranted.
